The article "Employing Atrous Pyramid Convolutional Deep Learning Approach for Detection to Diagnose Breast Cancer Tumors" was published in 2023. Journal: Comput Intell Neurosci.

# Employing Atrous Pyramid Convolutional Deep Learning Approach for Detection to Diagnose Breast Cancer Tumors

**DOI:** 10.1155/2023/7201479

**Published:** 2023-11-14

**Authors:** Ehsan Sadeghi Pour, Mahdi Esmaeili, Morteza Romoozi

**Affiliations:** Department of Electrical and Computer Engineering, Kashan Branch, Islamic Azad University, Kashan 8715998151, Iran

## Abstract

Breast cancer is among the most common diseases and one of the most common causes of death in the female population worldwide. Early identification of breast cancer improves survival. Therefore, radiologists will be able to make more accurate diagnoses if a computerized system is developed to detect breast cancer. Computer-aided design techniques have the potential to help medical professionals to determine the specific location of breast tumors and better manage this disease more rapidly and accurately. MIAS datasets were used in this study. The aim of this study is to evaluate a noise reduction for mammographic pictures and to identify salt and pepper, Gaussian, and Poisson so that precise mass detection operations can be estimated. As a result, it provides a method for noise reduction known as quantum wavelet transform (QWT) filtering and an image morphology operator for precise mass segmentation in mammographic images by utilizing an Atrous pyramid convolutional neural network as the deep learning model for classification of mammographic images. The hybrid methodology dubbed QWT-APCNN is compared to earlier methods in terms of peak signal-to-noise ratio (PSNR) and mean square error (MSE) in noise reduction and detection accuracy for mass area recognition. Compared to state-of-the-art approaches, the proposed method performed better at noise reduction and segmentation according to different evaluation criteria such as an accuracy rate of 98.57%, 92% sensitivity, 88% specificity, 90% DSS, and ROC and AUC rate of 88.77.

## 1. Introduction

Breast cancer occurs in the breast and has symptoms such as a lump in the breast, breast appearance changes, breast skin dimpling, nipple discharge other than breast milk, and/or flaky skin. Breast cancer is the second-most frequent cancer among women and causes a large number of deaths every year. It was reported that breast cancer is almost impossible to prevent since its causes remain unknown [1]. Therefore, early diagnosis is crucial in the treatment of breast cancer. Mammography is widely used by radiologists to diagnose and screen breast cancer. Today, mammography is the most commonly used technique for the early diagnosis of breast cancer and has reportedly lowered the mortality rate to 25%. However, it is difficult to interpret and describe mammographic images [2]. To obtain more accurate results, image preprocessing is required [1]. Preprocessing is primarily carried out to enhance image quality and improve diagnosis by removing unimportant segments from the background and to precisely extract breast areas by revealing breast boundaries [2]. The current mammography is based on smart medical diagnosis systems with image processing using machine learning (ML). Image processing principles in smart medical systems are important for the diagnosis of breast cancer since mammographic pictures are intrinsically noisy, which may challenge the diagnosis. In reference [3], a number of optimal filters have been introduced in order to detect sounds. Although intelligent diagnosis systems can remove noise and detect diseases, the judgment of doctors is necessary. Therefore, it is important to introduce an intelligent diagnosis system to diagnose breast cancer.

The article "Employing Atrous Pyramid Convolutional Deep Learning Approach for Detection to Diagnose Breast Cancer Tumors" was published in 2023. Journal: Comput Intell Neurosci.

In the proposed approach, a dataset called MIAS is used as the input dataset containing images and features of mammography for breast cancer diagnosis. This study is mainly based on image processing and deep learning techniques. In other words, an image is first used as the system input. It is then preprocessed through the quantum wavelet transform algorithm for noise reduction. Morphological processing is then performed with expansion, erosion, and border operators as well as segmentation operations for feature detection. Afterwards, the image and its features are used as the convolutional deep learning network input, and the windowing order is performed in the network by layering. Feature extraction is then presented with classification. The Atrous pyramid CNN was employed in order to prevent classification problems. The results indicated that the proposed approach improved the cancer type diagnosis accuracy as opposed to the most of previous methods. In this study, a morphology-based quantum wavelet transform approach was employed to improve and reduce noise. In fact, this quantum wavelet transform is among the wavelet transforms that operate faster in detecting noisy areas. Due to its quantum mode, this wavelet transforms benefits from a higher processing speed to detect any noise on mammography images. There are certain advantages and disadvantages to each of the previous papers and studies. For instance, most of them did not use real-time processing but had high computational complexities and long runtimes. Basically, they had an uncertainty structure, and their final diagnosis accuracies were lower than the results reported by this study, in which all of the aforementioned metrics were improved. In each research step, the proposed approach was compared with previous methods, something which indicated the superiority of the research results. In summary, this study presents a method based on image morphology operators for the segmentation of mammographic pictures with the goal of detecting the precise mass area.

The article "Employing Atrous Pyramid Convolutional Deep Learning Approach for Detection to Diagnose Breast Cancer Tumors" was published in 2023. Journal: Comput Intell Neurosci.

## 2. Literature Review

Since the intelligent diagnosis of breast cancer is a hot topic, numerous studies have been conducted using different methods in the literature. This section reviews the literature and the idea. This is classified into (1) breast tumor detection and classification, including the noise reduction of mammographic images, and (2) mammographic image diagnosis and classification.

### 2.1. Noise Reduction-Based Studies

The noise of mammographic images substantially affects image analysis and classification accuracy. Hence, it is important to reduce noise in mammographic images. The noise of a medical image is dependent on the imaging procedure. Mammographic images often have Gaussian, impulse (salt and pepper), and Poisson noises. Such noises should be minimized to avoid challenges in the next processing phase and breast tumor misdiagnosis.

#### 2.1.1. Salt and Pepper Noise

Salt and pepper noise appears in the form of corrupted white and black pixels, which could be sparse or dense. It is also known as impulse noise and often occurs in data transmission. Abrupt disruptions in the image signals are the main cause of salt and pepper noise. It has two scenarios of probability: zero or 255 (eight-bit images); it either makes a signal zero (destruction) or one (the noise replaces the signal) [4].

#### 2.1.2. Gaussian Noise

Gaussian noise, sometimes known as white noise, typically arises from electric sensors to capture image signals. It is based on the Gaussian distribution that is randomly selected and applied to the image. The Gaussian noise measure of a Gaussian distribution is given by

(1) $$\begin{array}{c} p\left(z\right)=\frac{1}{\sqrt{2\pi }\sigma }e^{\left({-\left(z-\bar{z}\right)}^{2}/{2\sigma }^{2}\right)}, \end{array}$$

where *z* is the gray level, $\bar{z}$ is the mean gray level, and *σ* is the standard deviation. Here, *z* and *σ* are the mean and variance of the Gaussian distribution, respectively [5].

#### 2.1.3. Poisson Noise

Poisson noise, also known as quantum mottle in medical physics, occurs in images due to Poisson processes. It arises from the distinct properties of photons. It appears between the original pixels in an image in a dispersed form. Poisson noise is found between the high-frequency components of an image [6].

A study on noise reduction from mammographic images [7] found that the level of noise significantly affected image analysis and classification. It is, therefore, important to reduce noise in mammograms. Medical images have different amounts of noise. Quantum noise is the most prevalent type of noise in mammography imaging. The goal of this research was to identify and investigate various filters in windows, including mean, middle, and Wiener filters of various sizes, using the DDSM (Digital Database for Mammography Screening) dataset. The greater the noise rating is, the higher the peak signal-to-noise ratio (PSNR) is, implying that the restored image has a higher image quality. The PSNR value was used to analyze the image quality of the restored filters. According to the results, for the reduction of noise in mammographic images, the 3 × 3 Wiener filter produced the best results.

The article "Employing Atrous Pyramid Convolutional Deep Learning Approach for Detection to Diagnose Breast Cancer Tumors" was published in 2023. Journal: Comput Intell Neurosci.

In another study [8], to reduce noise in grating-based mammographic images using X-ray, nonlocal denoising based on noise analysis was used. Noise analysis-based nonlocal denoising methods use noise variance similarity and dispersion to obtain the optimal weighted average using pixel intensity. The noise variance was calculated more accurately using a two-stage NLM-NANLM method. The method showed superb performance.

A study presented a preprocessing technique for mammograms using an adaptive weighted frost filter [9]. Mammography is the best successful technology for the initial detection of breast cancer in patients since it can identify cancer two years before symptoms appear. The pre- and postprocessing stages of the mammographic image identification procedure are computationally intensive. In all imaging approaches, initial processing is critical, with the most critical component being the implementation of techniques capable of enhancing the image's quality so that it can be used for further analysis and data extraction. This article discussed preprocessing, which is critical in mammographic picture analysis due to the low quality of mammography, which is taken at low doses since excessive radiation can threaten the patient's health. Numerous strategies have been developed to enhance image quality, smoothness, and noise restoration. The experimental results indicated that the suggested adaptive weight freeze filter is the optimal solution for noise reduction in mammographic pictures, outperforming other methods. The proposed technique was compared qualitatively and quantitatively to the other strategies available. The article's experiments demonstrated that the proposed strategy outperforms previous techniques.

In another study [10], the Bayes shrink (HMBS) method was introduced in order to reduce speckle noise in mammographic images. A combination of homogenous filters and downsized methods was used to reduce Bayes for denoising. Homogeneous filters were used to differentiate between homogenous areas and speckle noise, and seven criteria were employed to more accurately evaluate image quality.

The article "Employing Atrous Pyramid Convolutional Deep Learning Approach for Detection to Diagnose Breast Cancer Tumors" was published in 2023. Journal: Comput Intell Neurosci.

In reference [11], radiologists require high-quality and perfect mammographic images for more accurate diagnosis. Using convolutional neural networks (CNNs) as a deep learning model, a method for reducing noise in images and improving diagnosis was proposed. Poisson noise was increased, and ensemble transmission was used to convert it into white Gaussian noise. Moreover, the authors in [12] describe the development of an intelligent breast cancer detection system. This unique strategy is based on the use of image processing techniques to extract the tumor area while taking into account its significant characteristics. Then, seven features representing the tumor's texture and shape are retrieved and fed into a back-propagation neural classifier. The researchers also proposed the use of an interval type-2 fuzzy set and HM approach to fuzzify a breast cancer dataset [13]. They used the Wisconsin Breast Cancer dataset from the UCI data source for the purpose of creating the fuzzy breast cancer dataset. To overcome the limitations of the classic fuzzy type 1 method, the IT2 fuzzy models captured several expert opinions that addressed sharp boundary problems as well as inter- and intra-uncertainty among domain experts. By utilizing this database, rules and models will be developed that are more accurate.

### 2.2. Segmentation-Based Studies

Dissecting malignant masses in mammograms is a difficult task when there are issues such as low contrast, ambiguous, hazy, or divided boundaries, and the presence of severe abnormalities [14]. These facts exacerbate the difficulty of developing computer-aided diagnostics (CAD) tools to assist radiologists. The purpose of this article [14] was to offer a new mass separation algorithm for mammography based on robust multifunctional characteristics and automatic and maximal estimation (MAP). Four steps were proposed as part of the segmentation approach: a dynamic contrast enhancement strategy that applies to a specified region of interest (ROI), a technique for correcting background infiltration using matching templates, and mass candidate point recognition using posterior probabilities based on various scales.

The high degree of integration and the precise specification of the mass area are achieved through a MAP system in image segmentation. Segmentation was performed using 480 ROIs created in collaboration with two radiologists and ground truth. Three statistical criteria were utilized to assess its effectiveness in comparison with advanced segmentation techniques. The experimental results demonstrated that the created approaches are capable of comparing to other algorithms for ill-defined or thicker wastes. By incorporating it into a CAD system, radiologists may benefit from this strategy.

The article "Employing Atrous Pyramid Convolutional Deep Learning Approach for Detection to Diagnose Breast Cancer Tumors" was published in 2023. Journal: Comput Intell Neurosci.

The authors of [15] present a method for classifying and diagnosing breast cancer in mammographic pictures using a mix of wavelet analysis and a genetic algorithm. As presented in this paper, concerns have been raised about the reliability and sensitivity of detecting abnormalities in both lateral oblique and cranial-ear (CC) mammographic views. This study discussed a group of computational algorithms for identifying and segmenting mammograms with or without masses in the CC and MLO images. To begin, an algorithm for removing artifacts was run utilizing a wavelet transform and Wiener filter-based approach for gray-level enhancement. Additionally, a method has been presented for identifying and dividing masses randomly selected from the digital mammography screening dataset using genetic algorithms, multiple thresholds, and wavelet transforms genetic algorithms. An area overlap metric (AOM) was used to test the computer approach developed. Experiments demonstrated that the proposed method could be used to segment mammography masses in CC and MLO images. Additionally, this strategy overcame the examination of the CC and MLO representations.

Additionally, another study [16] proposed a semisupervised fuzzy GrowCut adaptive method of segmenting mammographic pictures based on the region of interest. In the study, the automaton evolution rule was modified to include a Gaussian fuzzy membership function in order to model undefined borders in a semisupervised version of the GrowCut algorithm. As part of this method, the manual selection of suspected lesion locations was replaced with an automated selection process that utilized a differential evolution algorithm only to select interior points. 57 lesion photos from the mini-MIAS database were used to assess this approach. The results were compared to those obtained using LBI, wavelet analysis, BMCS, BEMD, MCW semisurveillance, and the topographic technique. The results indicated that the method produced superior results for hybridized, thicker, and poorly acquired lesions due to the relation between the images of the grand tract and the segmentation results. In reference [17], using two fully convolutional neural networks (CNNs) based on SegNet and U-Net, two deep learning strategies were proposed for the automated segmentation of breast tumors in dynamic contrast-enhanced magnetic resonance imaging (DCE-MRI). The advantage and superiority of the proposed method in this study are its high accuracy in the division method for better and more accurate identification of the masses.

The article "Employing Atrous Pyramid Convolutional Deep Learning Approach for Detection to Diagnose Breast Cancer Tumors" was published in 2023. Journal: Comput Intell Neurosci.

In another study [18], earlier works developed a deep learning system to detect and diagnose breast cancer in mammographic images based on the end-to-end strategy. A transferable texture (TT)-CNN-based classification method was employed for cancer classification. The benign and malignant areas would be detected using the TT-CNN architecture once the mammographic images had been processed. Then, EL investigated the tissue features and extracted data from the image. For example, in reference [19], the U-net architecture was employed to segment fibroglandular tissue (FGT) and breast images. The model was demonstrated to substantially outperform other algorithms. A CNN was employed to segment mammographic images and find deep masses. In fact, a multipurpose segmentation was provided for different image areas. They demonstrated that an individual CNN architecture could be exploited to train other CNNs to obtain more accurate information from images using different methodologies [20]. For the segmentation of prostate and mammographic images, convolutional neural networks and deep learning have also been implemented. In this research [21], using the U-net model, breast lesions were segmented into two stages: U-net and quantity. The model was found to outperform other techniques and could be utilized for ultrasonic breast cancer detection and diagnosis. In another study [22], local adaptive thresholding and an advanced morphologic method were used for nuclear Allred cancer segmentation and classification in breast tissue images. They performed unsupervised classification of cancer nuclei. The model was calculated to have an accuracy of 98% in tumor-level measurement.

In reference [23], mammographic images were segmented to detect and classify cancerous tumor types (i.e., benign and malignant) from an optimal region growth perspective. The images would be noise reduction using a Gaussian filter prior to primary image processing. Drawing on the gray-level run length matrix (GLRLM) and gray-level co-occurrence matrix (GLCM) techniques on segmented images, tissue features were extracted and fed to a feed-forward neural network (FFNN). The tumors were classified into benign and malignant through a backpropagation (BP) algorithm. The model showed an accuracy of 97.8% and outperformed other models.

In [24], to detect and classify benign and malignant cancerous tumors, two automatic techniques were introduced: (1) the detection and classification of growing tumors, in which the threshold was obtained through a trained neural network, and (2) tumor detection and classification using a cellular neural network (CNN). The techniques were implemented on the mammographic image analysis society (MIAS) dataset, with the accuracy, sensitivity, and specificity being 95.94%, 96.87%, and 96.47%, respectively. A three-stage automatic system was proposed for the detection and classification of tumors using microarray images. The system was reported to have an accuracy of 95.45% [25]. An automatic backpropagation neural network (BPNN) model was introduced for the classification and detection of breast cancer tumors. It was reported to detect cancerous tumors with an accuracy of 70.4% [26]. The naïve Bayesian algorithm was adopted to detect and classify cancerous tumors on mammographic images. The accuracy, sensitivity, and specificity of the algorithm were reported to be 98.54%, 99.11%, and 98.25%, respectively [27]. In another study [28], a personal mammographic screening method was developed to diagnose cancer breast on mammographic images. It implemented screening decision-making based on the age of a patient. In reference [29], a hybrid predictor of breast cancer recurrence was employed. The model was calculated to have an accuracy of 85%. In reference [30], a hybrid of the firefly algorithm and artificial intelligence (AI) was employed to detect breast cancer. In another study [31], AI and image-processing techniques were employed to detect breast cancer. Furthermore, a new breast cancer detection methodology was introduced using ML algorithms. In reference [32], an automatic system was proposed for breast cancer classification. They used deep learning for the classification and detection of cancer on ultrasound images. The technique consisted of five phases: (1) data enhancement, (2) a pretrained model, (3) training the modified model through transfer learning (TL), (4) selecting the best features, and (5) the classification of the selected features using ML.

The article "Employing Atrous Pyramid Convolutional Deep Learning Approach for Detection to Diagnose Breast Cancer Tumors" was published in 2023. Journal: Comput Intell Neurosci.

In another study [33], bat-inspired algorithms (BA) can be utilized for cancer classification using microarray datasets for gene selection. Two stages are employed in gene selection, namely, the filter stage that utilizes the minimum redundancy maximum relevance (MRMR) method and the wrapper stage that utilizes BAs and SVMs. In this paper, the authors in [34] proposed a methodology to detect breast cancer and classify malignant and benign tumors. To extract features from mammogram images, ML and hybrid thresholding were employed. The model was evaluated on four mammogram image datasets, including MIAS, DDSM, INbreast, and BCDR. The model was found to show maximum performance on the MIAS dataset.

In reference [35], a new feature learning approach was proposed to detect and classify breast cancer using an artificial neural network (ANN) with optimized hidden layers. The classification sensitivity, accuracy, and specificity were reported to be 0.9815, 0.9948, and 0.9882, respectively. In this review [36], earlier works reviewed the literature on kidney cancer detection and the classification of malignant and benign tumors using ML and deep learning algorithms. In reference [37], the literature on breast cancer detection and classification based on ML algorithms was reviewed. The detection of breast cancer on mammographic images is carried out in three stages: (1) image preprocessing, (2) feature extraction, and (3) classification and evaluation. A total of 93 works were reviewed, reporting that deep learning techniques account for the majority of the effective methods that are used for cancer detection.

## 3. Proposed Method

The present study primarily aimed to implement the early detection of breast cancer on mammographic images and tumor classification into benign, malignant, and suspicious using a hybrid of image processing techniques and deep learning.  Figure 1 demonstrates the proposed method diagram in which the operations of each step are presented briefly.

The proposed approach consists of three major steps, the first of which includes preprocessing to improve and reduce noise on mammography images through the quantum wavelet transform. In the second step, morphological processing is used for image segmentation. In fact, these two steps are considered the phase of image processing and machine vision. The third step operates with a deep learning structure based on an Atrous pyramid convolutional neural network (APCNN) that actually selects and extracts features in addition to performing classification operations to diagnose benign, malignant, and suspicious cases of cancer. It can also pinpoint the accurate locations of cancerous tumors on an image. This step belongs to the machine learning phase.

### 3.1. Preprocessing Phase

The input images should be normalized. In the preprocessing phase, mammographic images were normalized as input data (often noisy) and were improved to enhance system efficiency. The image is changed to a predefined size and reasonably filtered using quantum wavelet transform. Then, the input data are normalized. A two-dimensional array of pixels in the range [0, 225] is used to display individual images in a hybrid of local thresholding and active contours. The local thresholding process initializes images in two stages. It is assumed that the noisy input image will be the initial image for denoising. This is carried out by local search operators to improve the initial pictures using quantum wavelet transform. Therefore, following the first phase, a deconstructed image will exist. The second stage involves thresholding the detail coefficients and randomly selecting one of these decomposed regions for reconstruction. The following definitions apply to the reconstruction section:

- Gauss fading: filter image using a Gaussian filter
- Means filter: filter image using a mean filter
- Change in intensity: a similar criterion is chosen at random between [0.7, 1.3] to multiply all picture pixels
- Adaptation of light intensities: an inverse quantum wavelet transform filtering technique based on quantum and inverse processing is used to construct the quantum inverse structure

The following steps will then be taken:

- One-point row: randomly selected pixels in a row
- One-point column: randomly selected pixels in a column
- Point-to-point pixel: as each pixel disappears, it is replaced by a random pixel
- Classifying all the points as rows and columns in the pictures and diagonally to decrease the noise in quantum wavelet transform

In the quantum wavelet transform filtering algorithm, a new picture may be passed through the local search operator when the selection value is less than the range [0, 1] lower than the local search rate. Each pixel in the image is sorted by its pixel value after the decomposition process has been completed, and the best coefficients are used as quantum values for the operation at hand. There are several ways to decompose a signal in mammographic pictures into several displaced or scaled displays of previously extracted characteristics. In order to break down an image into its constituent components, local thresholding and active contours can be applied. After applying the quantum wavelet transform, local thresholding, and active contours, the image is segmented. Some details can be eliminated by applying quantum wavelet transform-based local thresholding and active contour coefficients. Local thresholding and QWTF based on active contour provide the significant advantage of distinguishing small features in an image. It is possible to isolate very small details in an image using active contours, while larger details can be detected using local thresholding. The combination of small and large details and reading all rows and columns linearly and diagonally meet the quantum wavelet transform structure so that mammographic image noise can be minimized. Two characteristics are present in a local thresholding-active contour function with quantum wavelet transform. First, it is a vibrational function or has a wave-like form, such as follows:

(2) $$\begin{array}{c} \int_{-\infty }^{0}\Psi \left(t\right){|}^{2}dt<\infty . \end{array}$$

The maximum energy in Ψ(*t*) occurs in a limited period, which is written as follows:

(3) $$\begin{array}{c} \int_{-\infty }^{0}\Psi \left(t\right)dt=0. \end{array}$$

Reducing the noise method is written as follows:

(4) $$\begin{array}{c} \text{Method}\left(I\right)=\left(\underset{\Omega }{\sum }\sqrt{1+\alpha^{2}|\nabla I{|}^{2}}\right)+\frac{\gamma }{2}{\left(I-I_{0}\right)}^{2}. \end{array}$$

In this function, the image edges are taken into account, and important characteristics of the image are preserved. The term (*I* − *I*_0_)^2^ ensures a specific degree of validity between the picture under evaluation and the original picture, in which *I* and *I*_0_ represent the picture under study and the original picture, respectively. Furthermore, ∇*I* is the total diversity tuning period, *α* and *γ* are balancing parameters, and *Ω* is the total of pixels in the picture. The minimization of equation (3) reduces the total picture diversity while preserving validity. Overall, input data are normalized in the preprocessing phase and improved, if needed, to enhance the detection performance of the system.

The article "Employing Atrous Pyramid Convolutional Deep Learning Approach for Detection to Diagnose Breast Cancer Tumors" was published in 2023. Journal: Comput Intell Neurosci.

It is important to note that by adjusting the sum of the variations ∇*I*, a mammography picture may have some noise such as salt and pepper, Gaussian, or blur effects. Therefore, this variation was used to determine the types of this noise variation and to calculate its sum. In this article, QWTF is proposed as an innovative noise reduction method for mammography. Earlier works adopted the matched filter technique to introduce a strategy to detect macroscopic dark material objects in images [38], and also, a quantum image filter in the frequency domain was introduced based on the Fourier transform [39]. It should be noted that the threshold value was determined by trial and error.  Figure 2 illustrates how to identify noisy pixels.

For identifying noisy pixels in figures, each pixel has four brightness values ranging from white to black, and these values are pos=*|*01> and color=*|*10> for dark gray, pos=*|*00> and color=*|*01> for gray color, Pos=*|*11> and color=*|*11> for white color, and Pos=*|*11> and color=*|*11> for black color.

### 3.2. Image Segmentation Phase

The segmentation of images is one of the most important and complex parts of image processing and computer vision. Today, segmentation is a standard image processing and manipulation process in many software packs and systems. In this process, similar pixels are segmented into the same class. In other words, images are partitioned into sections or objects. To effectively identify the image space, it is required to identify the foreground and background. To this end, internal edge detection is used, and different segments of an image can be separated in terms of color and light based on edges. The input of the segmentation phase consists of images that have been denoised and improved in the preprocessing phase. The operation is carried out based on the morphology in the segmentation phase. This algorithm is used for two reasons. First, an image is assumed to be a search space, and segmentation can be used to improve the search space. This effectively reduces dimensionality, extracts features, and implements classification to enhance performance. Second, it boosts the speed and convergence of image processing and avoids local optimal. It is worth mentioning that edge detection based on the Sobel operator is also utilized. In this respect, MATLAB has preprocessing instructions.

The article "Employing Atrous Pyramid Convolutional Deep Learning Approach for Detection to Diagnose Breast Cancer Tumors" was published in 2023. Journal: Comput Intell Neurosci.

Mathematical morphology helps extract image components, which is very useful for describing segment features and shapes, such as frameworks, convex shells, and boundary areas. The mathematical morphology language is set theory, and morphology is a powerful, unified technique to cope with image processing problems. Here, sets represent objects in an image. Erosion and dilation are the two essential operations in morphological image processing. A segmentation phase is performed to segment mammographic images using morphology based on erosion and dilation operations and boundary extraction. Let *M* and *v* be sets in *q*. The erosion of *M* and N is written as follows:

(5) $$\begin{array}{c} M\;⊖\;N=\left\{Q|{\left(B\right)}_{q}\subseteq M\right\}. \end{array}$$

The erosion of *M* and *N* is a set of all points of *q* such that *N* transferred by *q* is located in *M*. *N* is assumed to be a structuring element =. Since *N* should be in *M*, set *N* and the background share no objects. Erosion can also be formulated as follows:

(6) $$\begin{array}{c} M\;⊖\;N=\left\{Q|{\left(N\right)}_{q}\cap M^{c}=\emptyset \right\}, \end{array}$$

where *M*^*c*^ is the complement of *M* and ∅ is the empty set. Let *M* and *N* be set in *Q*^2^. The dilation of *M* and *N* is written as follows:

(7) $$\begin{array}{c} M\;⊕\;N=\left\{Q{\left(\overset{\wedge }{N}\right)}_{q}\cap M\neq \emptyset \right\}, \end{array}$$

where dilation is implemented by reflecting *N* around its origin and transferring the reflection by *q*. Then, the dilation of *M* by *N* is the set of all movements in *q* such that $\overset{\wedge }{M}$ and $\overset{\wedge }{N}$ have at least one common element. Therefore, dilation is formulated as follows:

(8) $$\begin{array}{c} M\;⊕\;N=\left\{Q|\left[{\left(\overset{\wedge }{N}\right)}_{q}\cap M\right]\subseteq M\right\}. \end{array}$$

Based on equation (8), *N* is a structuring element and *M* is a set of image objects to be dilated. The boundary of set *M*, shown as *β*(*M*), can be found by eroding *M* by *N* and subtracting *M* from its erosion as follows:

(9) $$\begin{array}{c} \beta \left(M\right)=M-\left(M\;⊝\;N\right). \end{array}$$

Based on equation (9), *N* is a suitable structuring element.

The article "Employing Atrous Pyramid Convolutional Deep Learning Approach for Detection to Diagnose Breast Cancer Tumors" was published in 2023. Journal: Comput Intell Neurosci.

For calculating the fitness function of *f* in the proposed image morphology operators in this article, the dataset considers as *R*_*N*×*D*_ which *N* is the sample from per image and *D* is the sample's distance (features) which will have *K* segmented parts and *f* calculated as follows [40]:

(10) $$\begin{array}{c} f=\text{minimize}\overset{N}{\underset{i=1}{\sum }}\overset{K}{\underset{m=1}{\sum }}{\left[\delta \left(r_{i,d},c_{m,D}\right)\right]}^{2}. \end{array}$$

In this equation, *δ* is distance (features) metric as Euclidian between any segmented parts which is defined based on two features: brightness and edges.

### 3.3. Atrous Pyramid CNN

This section presents APCNN based on convolutional neural networks as a new method of deep learning that can simultaneously calculate features and classify data. However, for the purpose of this research, it is intended that it would be able to determine breast cancer and then to identify the exact area of the masses followed by classifying them into malignant, benign, and suspicious classes. This section will be called APCNN which optimizes CNN with Moore–Penrose matrix and also CNN with this matrix. There are two general disadvantages associated with most neural network structures that can be addressed by adjusting the weights in the training phase using the descending gradient, as well as the volume of training data, in contrast to the classic CNN method. A further weakness in neural networks is a slowdown in the training process. This weakness can be resolved quickly during the training and testing phases, which is abundant after considerable data have been gathered. Neural networks also do not have the capability to train and test the same data if a similar dataset is imported or new data is entered into the same dataset which is another weakness of neural networks that is named generalization. Thus, there are many different types of neural networks that cannot be generalized. For this study, we will focus initially on CNNs.

It is interesting to note that in this study, the CNN will be optimized as an APCNN so that it can be run rapidly with generalizability and that is a result of the difficulties associated with neural network structures. As a result of its high learning speed and ability to adjust a parameter during the training phase as opposed to adjusting a number of parameters during the training phase in neural networks, this algorithm is often used. One of the major disadvantages of CNN is its inability to perform normal extraction, feature extraction, and classification operations. However, it will be performed by optimizing CNN and building APCNN structures. A CNN is a neural network that involves the input layer attached to a series of weights for the hidden layer, which are initially assigned a random value and are not reset during the training process, which is time-consuming. Unlike conventional neural networks, CNN uses normal neurons in the hidden layer; therefore, it does not require centroids and sigmas. Finally, there is only one parameter that needs to be adjusted in the CNN: synaptic weights between hidden and output layers. A typical CNN is a feed-forward structure that calculates synaptic weights in real time using an inverse pseudostructure, resulting in faster data training and testing. The overall architecture can be seen in Figure 3.

The article "Employing Atrous Pyramid Convolutional Deep Learning Approach for Detection to Diagnose Breast Cancer Tumors" was published in 2023. Journal: Comput Intell Neurosci.

The most important reasons for using CNN in this study instead of other smart methods in the classification and feature extraction phase are shown in Table 1.

CNN, in general, can be viewed as the exact opposite of deep learning methods and other classification methods such as naive Bayesian and SVM methods. Due to the algorithm's tremendous flexibility, it can use nonlinear activation functions such as sinusoidal, sigmoid, or nonderivative activation functions in addition to linear activation functions to neurons or activate cells in the hidden layer. By default, CNN has an equation in the general mode such as follows:

(11) $$\begin{array}{c} z\left(p\right)=\overset{m}{\underset{j=1}{\sum }}{\beta_{i}\beta }_{j}g\left(\overset{n}{\underset{i=1}{\sum }}w_{i,j}x_{i}+b_{j}\right). \end{array}$$

According to this equation, *β*_*i*_ represents the weights between the input layer and the hidden layer, and *β*_*j*_ represents the weights between the output layer and the input layer. *b*_*j*_ is the threshold value of neurons in the hidden layer, or bias. *g*(…) is the transition or actuator function. *w*_*i*,*j*_ is the input layer weights, and *b*_*j*_ is the bias that are assigned at random. At the start of the number of input layer, neurons, *n*, and hidden layer neurons, *m*, the activation function *g*(…) is assigned. According to this knowledge, if the known parameters for overall balance are merged and calibrated, the output layer will resemble as follows:

(12) $$\begin{array}{c} H\left(w_{i,j},b_{j},x_{i}\right)=\left[\begin{array}{c} g\left(w_{1,1}x_{1}+b_{1}\right)\\ g\left(w_{n,1}x_{n}+b_{1}\right) \end{array}\begin{array}{c} \ldots \\ \ldots \end{array}\;\begin{array}{c} g\left(w_{1,m}x_{m}+b_{m}\right)\\ g\left(w_{n,m}x_{m}+b_{m}\right) \end{array}\right],\;andz=H\beta . \end{array}$$

The main goal in all models of training-oriented algorithms is to minimize the error whenever possible. *z*_*p*_ is a function that outputs errors obtained by the actual output *z*_main_ in CNN, which can be represented by two training sections, namely, ∑_*k*_^*s*^(*z*_main_ − *z*_*p*_) and testing sections, namely, ‖∑_*k*_^*s*^(*z*_main_ − *z*_*p*_)^2^‖. For both functions, the output *z*_*p*_ obtained by the actual output *z*_main_ must be equal to *z*_*p*_. An unknown parameter is specified when this equation is executed, and the results are satisfied. The matrix *G* can be a matrix that is very unlikely. As a result, there may be a discrepancy between the whole number of attributes in the training and those in the test set. Therefore, inverting [*G*] and locating weights are important issues. CNN overcomes this challenge by using a matrix referred to as Moore–Penrose, which can be used to develop approximate inverse matrix computations that are capable of performing dimensionality selection and feature extraction operations with classification with increased accuracy and speed in comparison to other methods. Using the Moore–Penrose matrix, *α*^*∗*^ is the output matrix and *G*^*∗*^ is the generalized inverse Penrose matrix of *G*. Thus, due to the optimization of the CNN, the problem of output weights in the CNN was solved as *A*^*∗*^=*G*^*∗*^ which became the APCNN or Moore–Penrose matrix extreme learning machine. Generally, APCNN becomes a chain of repeating modules over time in the training phase. APCNN will be able to work like a conveyor that is to add or subtract information from neurons. APCNN does not require weight updating during training, unlike deep learning structures or other classification models such as naive Bayesian models and support vector machines. Unlike deep learning structures and other classification models, such as support vector machines or naïve Bayesian, no weight update operations are performed during training. APCNN can specify attributes at the intersection. By minimizing APCNN energy performance, a suitable model is taught that can be modeled as follows:

(13) $$\begin{array}{c} E\left(Y\right)=\overset{N}{\underset{i}{\sum }}\Psi_{v}\left(y_{i}\right)+\overset{N}{\underset{\forall i,j,i\neq j}{\sum }}\Psi_{q}\left(y_{i},y_{j}\right). \end{array}$$

In this case, *v*, *q* ∈ {1,2,…, *C*_*n*_) are the intersection labels, and *i*, *j* ∈ {1,2,…, *N*} are specific pixels of the original image or *I*. Ψ_*q*_(*y*_*i*_)=−log *P*(*y*_*i*_*∣I*) is a negative logarithmic probability in which *P*(*y*_*i*_*∣I*) is a probability calculated by the APCNN algorithm for each pixel I. As part of the evaluation of two APCNN matrices in a fully connected layer, it is necessary to examine the relationship between each pair of pixels outlined in the following equation:

(14) $$\begin{array}{c} \Psi_{q}\left(y_{i},y_{j}\right)=\eta \left(y_{i},y_{j}\right)\overset{N}{\underset{n=1}{\sum }}w^{\left(n\right)}k^{\left(n\right)}\left(f_{i},f_{j}\right). \end{array}$$

In this equation, *N*=2 is the number of Gaussian core and *w*^(*n*)^ indicates a weight for the *m*th Gaussian core. *η*(*y*_*i*_, *y*_*j*_)=[*y*_*i*_ ≠ *y*_*j*_] is the consistent function tag. *k*^(1)^ demonstrates the appearance of the core appearance, which attempts to assign the same class tags to adjoining and similar intensity pixels adjacent to each other. *k*^(2)^ demonstrates the core smoothness, which is connected with the objective of removing superfluous parts. Overfitting and data redundancy may occur within the max-pooling layer in matrix convolution deep learning. Generally, these problems are common in neural networks, especially in matrix convolution deep learning. Hence, matrices were used in this study to prevent these problems and accelerate training and testing for the detection and extraction of features. These two steps are denoted by equations (15) and (16), respectively.

(15) $$\begin{array}{c} k^{\left(1\right)}\left(f_{i},f_{j}\right)=\exp\;\left(-\frac{\left|s_{i}-s_{j}\right|}{2\theta_{\alpha }^{2}}-\frac{\left|e_{i}-e_{j}\right|}{2\theta_{\beta }^{2}}\right., \end{array}$$

(16) $$\begin{array}{c} k^{\left(2\right)}\left(f_{i},f_{j}\right)=\exp\;\left(-\frac{\left|s_{i}-s_{j}\right|}{2\theta_{\gamma }^{2}}\right). \end{array}$$

*e*_*i*_ and *e*_*j*_ are the light intensities of the pixels *i*, *j*, *s*_*i*_, and *s*_*j*_ of the corresponding spatial coordinates. *f*_*i*_ and *f*_*j*_ display the characteristics of each pixel pair, i.e., the brightness intensity and spatial information. *θ*_*α*_, *θ*_*β*_, and *θ*_*γ*_ show the parameters of the Gaussian cores, respectively. However, some points may not be cut in this way; therefore, an optimization of this algorithm will be done in layers. Generally, the layers of the APCNN method are employed by using the input layer with the number of neurons. As part of the training and testing layer, convoluted layers, pooling layers, and fully connected layers have been implemented along with Moore–Penrose. Next, a soft-max layer and an output layer are then embedded in order to display the results. Matrix-based windowing is used for the training layers as measured by 9 × 9 in the convolve layer, 7 × 7 in the random pooling layer, and 5 × 5 in the maximum pooling layer. The fully connected layer's structure is CRF, and its window structure is 9 × 9. The soft-max layer is also 7 × 7. As part of the initial APCNN training and segmentation process, convolve and pooling layers are sequentially inserted into the training layer, which consists of a convolve layer, a random pooling layer, another convolve layer, and finally a maximum pooling layer. There is a completely connected APCNN layer at the conclusion of this training layer. Then, outside the training layer, there is a soft-max layer, which is used to optimize specification operations and motion object tracking following feature extraction using the probabilistic particle filtering technique. It is important to keep in mind that the amount of neurons in each segment is critical. For every convolve and pooling layers, there are seven Atrouses (*r*). In order to enhance the segmentation and feature extraction activities during the training of the deep neural network of the soft-max layer, the APCNN method is applied. The state of a dynamic system can be approximated using Bayesian filters based on a sequence of sensory observations with noise. To begin, the most widely known Bayesian rule is that a probability for an APCNN technique is eliminated (thus, the name Atrous pyramid), whose model is the following equation:

(17) $$\begin{array}{c} p\left(C|D\right)=\frac{p\left(D|C\right)\times p\left(C\right)}{p\left(D\right)}. \end{array}$$

If Bayesian procedures are used to update the H assumption under the premise of *E* and *I*, there is the following equation:

(18) $$\begin{array}{c} p\left(H|K,L\right)=\frac{p\left(K|H,L\right)\times p\left(H|K,L\right)}{p\left(K|L\right)}. \end{array}$$

In this case, *p*(*K|H*, *L*) is the likelihood of the subsequent occurrence of *H* assumption based on the assumption of observing *E* in test conditions *L*. *p*(*H|K*, *L*) indicates the likelihood that the *H* assumption will take place prior to the *L* test conditions and the *E* perspective. Rate of similarity *p*(*H|K*, *L*) indicates the likelihood that the *K* assumption will occur when the *H* hypothesis meets the *L* test conditions and, lastly, the *p*(*K|L*) criterion for homogenization. When all measurements and values are taken into account, it is assumed that *S*(*m*) up to and including *m* and the value of *R*(*m*) of a dynamic system at *m*th can be predicted. Alternatively, a probabilistic probability can be calculated using a Bayesian formula:

(19) $$\begin{array}{c} p\left(R\left(m\right)|S\left(m\right)\right), \end{array}$$

so that *S*(*m*)={*s*(1), *s*(2),…, *s*)*m*)} is the set of all observations, and similarly, the state set of values *R*(*m*) is defined as *R*(*m*), and *R*(0) contains historical information about the system's status (before any observation). Bayesian rules thus become a type of the following equations:

(20) $$\begin{array}{c} p\left(R\right.\left(m\right)|S\left(m\right)=\frac{p\left(S\left(m\right)|R\left(m\right),S\left(m-1\right)\right)\times p\left(R\left(m\right)|S\left(m-1\right)\right)}{p\left(T\left(n\right)|S\left(m-1\right)\right)}, \end{array}$$

(21) $$\begin{array}{c} p\left(R\left(m\right)|S\left(m\right)\right)=W\left(m\right)\times p\left(S\right.\left(m\right)\left|R\left.\left(m\right)\right)\times p\left(R\right.\left(m\right)\right|S\left(m-1\right), \end{array}$$

(22) $$\begin{array}{c} p\left(R\right.\left(m\right)|S\left(m-1\right)=\int p\left(R\right.\left(m\right)\left|R\left(m-1\right)\times p\left(R\right.\left(m-1\right)\right|S\left(m-1\right)dr\left(m-1\right). \end{array}$$

In these relationships, *p*(*R*(*m*)*S*(*m*)) is a new estimation, *W*(*n*) is scaling, *p*(*S*(*m*)*∣R*(*m*)) are probably observations of a motion object, and *p*(*R*(*m*)*∣S*(*m* − 1) is the probability before observing the tumor masses based on sentinel lymph nodule, metastasis, and assessment of mitotic density. Also, *p*(*R*(*m* − 1)*∣S*(*m* − 1) is the preceding estimation, and *p*(*R*(*m*)*∣R*(*m* − 1) is system dynamics in the detection of tumor masses. Now, assuming that the *S*(*m*) are independent of one another, the system is described as a probabilistic APCNN process. By and large, the proposed Bayesian models are quite intricate, and it is difficult to study Gaussian distributions, at least in terms of linear models. While relationships can be simplified to achieve the required level of deep learning, generally, in order to solve equations, probabilistic APCNN techniques are used to consider all possible variations.

The article "Employing Atrous Pyramid Convolutional Deep Learning Approach for Detection to Diagnose Breast Cancer Tumors" was published in 2023. Journal: Comput Intell Neurosci.

Probabilistic APCNN has as its primary objective to determine the conditional density probability function for the mode vector and the measurement vector, and to apply Bayesian theory without utilizing any linearization and just modeling the entire system dynamically. This is one of the Monte Carlo statistical approaches, whereby the distribution function corresponds to the conditional probability of the weighted sum of a number of discrete functions. There are several types of Bayesian filters, which are commonly referred to as Bayesian bootstrap filters. Bayesian filters enable the estimation of a mode vector element's function based on the minimum error variance. Apart from Bayesian concerns and theory, as a result of equation (23), the method particles are defined as probabilistic for use in the soft-max layer of the APCNN algorithm; it is a function of the normal distribution function in two-dimensional and three-dimensional spaces.

(23) $$\begin{array}{c} p\left(\bar{x}\right)=\frac{1}{2\pi \sigma_{1}\sigma 2_{2}}e^{-\left[{\left(x_{1}-\mu_{1}\right)}^{2}/2\sigma_{1}^{2}+{\left(x_{2}-\mu_{2}\right)}^{2}/2\sigma_{2}^{2}\right]}. \end{array}$$

APCNN can also identify and classify data into three categories: benign, malignant, and suspicious cancers.

## 4. Simulation and Results

A MATLAB platform was used for simulation and analysis. A statistical analysis of the MIAS dataset has been used in this study. The characteristics of the data used in the MIAS dataset are clump thickness, uniformity of cell size, uniformity of cell shape, marginal adhesion, single epithelial cell size, bare nuclei, bland chromatin, normal nucleoli, and mitoses. Based on the statistical data of this section, we will be able to accurately diagnose breast cancer, nonbreast cancer, and suspicious cases in this dataset. We may download this dataset at https://peipa.essex.ac.uk/info/mias.html link, which contains seven columns, as shown in Table 2:

The simulation is created step by step. As shown in Figure 4, when the simulation begins, the input image is executed and displayed.

As part of the preprocessing process, the first step is to reduce the picture size and make it identical with the original noise reduction by using a simple median filter to reduce noise. To reduce noise and improve the picture, the proposed quantum wavelet transform filtering method is then used, as shown in Figure 5.

According to statistical analysis, the proposed noise reduction approach has high capabilities in comparison to previous methods; Table 3 illustrates the evaluation criteria by case.

By pressing the segmentation with the image morphology operator button, the social spider algorithm performs the segmentation operation at a speed of 0.5 seconds, as shown in Figure 6.

It is necessary to define operators of the social spider algorithm segmentation algorithm for the initial population of spiders with 100 spiders, the blade vibration rate of 2 as standard, and the rate of prey attack as 0.02 as standard and to take into account the initial presentation of the algorithm as well. Segmentation is performed at 100 iterations, using both color and edge properties. On the basis of statistical analysis, the proposed algorithm has a high capability when compared with previous approaches to image segmentation.  Table 4 shows a comparison of this approach to other methods in terms of evaluation criteria.

The article "Employing Atrous Pyramid Convolutional Deep Learning Approach for Detection to Diagnose Breast Cancer Tumors" was published in 2023. Journal: Comput Intell Neurosci.

Subsequently, the morphology-based quantum wavelet transform algorithm was employed with the boundary operator for noise reduction in the segmentation stage. The noise was reduced as much as possible for the accurate zone detection and final classification, and Figure 7 depicts the output.

The deep convolutional neural network (CNN) is then used for two purposes: feature extraction and final classification. Therefore, the pyramid deep CNN is employed for feature extraction including dimensionality reduction and feature selection. Moreover, the Atrous deep CNN is utilized to classify and indicate masses accurately within a spectrum in the image. In fact, the pyramid CNN should be adopted for dimensionality reduction, feature selection, and feature extraction based on the training and test models, in which 70% and 30% of data are used for training and test methods, respectively. There is a general output shown in Figure 8 that indicates only the breast. These operations are performed with the features introduced in Table 2 such as the column thickness, cell size uniformity, cell shape uniformity, marginal adhesion, single epithelial cell dimensions, naked cores, long chromatin, normal cores, mitosis, brightness, and edges. Furthermore, these features are used for the main research purpose that is to diagnose the metastasis of sentinel lymph nodes and assess mitotic density.

The classification operations are then performed by defining three classes (i.e., benign, malignant, and suspicious) and displaying the areas of cancerous tumors in mammography images, and Figure 9 indicates the output.

The operations in an input image have been displayed. However, all outputs should be implemented on a complete MIAS dataset. For this purpose, it is necessary to classify the analytical and statistical data of MIAS, which will be performed through the Atrous pyramid CNN. This method is adopted due to its simplicity among neural networks with a high convergence rate in training. However, it has some defects that can be covered with moving functions in addition to using a training core and the Atrous approach. Moreover, 70% and 30% of statistical data and images of MIAS were used for training and test methods, respectively. The Atrous pyramid CNN has nine major inputs with 10 hidden layers in the first layer and 2 hidden layers in the second layer. It also has two outputs called the detection of a tumor or mass in the breast or its absence. However, the third case known as the suspicious state was considered separately. If the output indicates neither the presence nor the absence of a tumor or a mass in the breast, it will be considered suspicious. Figures 10–13 demonstrate the efficiency, training modes, confusion matrix, and ROC of the Atrous pyramid CNN, respectively, and for breast cancer diagnosis based on MIAS images. Moreover, the ROC was used as the validation method along with K-fold and AUC.

The article "Employing Atrous Pyramid Convolutional Deep Learning Approach for Detection to Diagnose Breast Cancer Tumors" was published in 2023. Journal: Comput Intell Neurosci.

Figure 14 depicts another diagram showing the accurate results of classification. This can be used to accurately diagnose breast cancer based on mammography images.

The 5 K-fold validation method was employed to draw outputs in Figure 14. It is evident that our method provides good results in the classification phase. 98.57% accuracy was obtained in this method.  Table 5 reports the evaluation criteria for the proposed Atrous pyramid CNN. On the other hand, Table 6 shows the results of comparing this method with previous methods. The entire proposed approach should be represented as a ROC diagram from the beginning, i.e., preprocessing, segmentation, and then feature extraction and classification operations, and the output is in the form of Figure 15.

The final output, which completely extracts and displays the lesion or mass, is shown in Figure 16.

## 5. Discussion

Since medical diagnosis systems require reliable and fast methods to ensure doctors, it is essential to use smartification principles in developing such systems. Moreover, developing smart medical diagnosis systems can reduce human errors and help doctors diagnose diseases. As a result, the early diagnosis will help determine people's health status and provide them with further care until full recovery. Forming in different areas of the body, cancerous tumors do not have regular shapes and specific patterns. Imaging various areas of the body can help detect cancerous areas and determine the dimensions of these tumors. Medical principles can also be employed to estimate benign and malignant tumors. In fact, it is necessary to diagnose these tumors as accurately as possible, for they are among the most important causes of death all over the world. Thus, smart systems must be developed inevitably. Due to budget and time constraints in this study, we were unable to test the proposed approach on other datasets. Other research constraints included lacking powerful systems for data processing. A totally ordinary system was used in this study. Its specifications were already mentioned.

## 6. Conclusion

The early diagnosis of breast cancer helps prevent the growth of malignant tumors. Thus, it is necessary to develop an intelligent diagnosis model in order to reduce human errors and accelerate cancer diagnosis. This study proposed a novel technique to detect breast cancer on mammographic images and classify benign, malignant, and suspicious tissues. The MIAS dataset consisting of mammographic images and features in breast cancer detection was employed. The proposed model is based on image processing and deep learning. The input system is introduced to the system and preprocessed using the quantum wavelet transform algorithm to reduce noise. Then, morphological image processing is carried out through erosion and dilation operations and boundary extraction to implement segmentation and identify features. Then, image improvement is performed through the quantum wavelet transform algorithm. The features and image are fed as input to the CNN, and windowing is performed through layering. Then, the extracted features and classification are provided. To handle the classification challenges of pyramid CNNs, an Atrous CNN was employed. The proposed approach was found to outperform earlier methodologies in noise reduction and image segmentation. It had also a better receiver operating characteristic (ROC) curve and a larger area under the ROC curve (AUC). The accuracy, sensitivity, specificity, and DSS of the proposed model were obtained to be 98.57%, 92%, 88%, and 90%, respectively. Furthermore, the AUC rate and ROC were calculated to be 88.77%.

The article "Employing Atrous Pyramid Convolutional Deep Learning Approach for Detection to Diagnose Breast Cancer Tumors" was published in 2023. Journal: Comput Intell Neurosci.

## Figures and Tables

**Figure 1:** Proposed method diagram.

**Figure 2:** Identifying noisy pixels [38].

**Figure 3:** CNN's main architecture.

**Figure 4:** Input image.

**Figure 5:** Noise reduction with QWTF.

**Figure 6:** Image segmentation with morphology.

**Figure 7:** Noise reduction after segmentation.

**Figure 8:** The feature extraction output of the pyramid deep CNN.

**Figure 9:** An area of a cancerous tumor in the spectral images of the breast through Atrous pyramid CNN.

**Figure 10:** Classification efficiency of Atrous pyramid CNN.

**Figure 11:** Training modes of classification with Atrous pyramid CNN.

**Figure 12:** Confusion matrix of classification with Atrous pyramid CNN.

**Figure 13:** ROC of classification with Atrous pyramid CNN.

**Figure 14:** Accurate results of classification.

**Figure 15:** AUC and ROC curves for the overall results of the proposed approach.

**Figure 16:** Sample for the detection of cancerous masses at the end of the process.

**Table 1:** Comparison of APCNN with other conventional intelligent methods.

Naïve Bayesian	Support vector machine (SVM)	Extreme learning machine (ELM)	Recursive neural network (RNN)	Convolutional neural network (CNN)	APCNN
Training process is slow	Training process is slow	Training process is slow	Training process is slow	Faster training process	Faster training process
Binary classification ability	Binary classification ability	Multiclass classification ability	Multiclass classification ability	Multiclass classification ability	Multiclass classification ability and multiobjective and real time
Quadratic programming	Quadratic programming	Nonlinear multiobjective programming	Multiobjective quadratic programming	Nonlinear multiclass	Nonlinear multiclass and multiobjective programming

The article "Employing Atrous Pyramid Convolutional Deep Learning Approach for Detection to Diagnose Breast Cancer Tumors" was published in 2023. Journal: Comput Intell Neurosci.

**Table 2:** The information available in the MIAS dataset.

#1	#2	#3	#4	#5	#6	#7
MIAS database reference number	Character of background tissue: F, fatty G, fatty-glandular D, dense-glandular	Class of abnormality present: CALC, calcification CIRC well-defined/circumscribed masses SPIC, spiculated masses MISC, other, ill-defined masses ARCH, architectural distortion ASYM, asymmetry NORM, normal	Severity of abnormality; *B*, *benign* M, malignant	*x*, *y* image coordinates of center of abnormality	*x*, *y* image coordinates of center of abnormality	Approximate radius (in pixels) of a circle enclosing the abnormality

**Table 3:** Comparison of noise reduction approach in this research with previous methods.

References	Noise reduction approach	Windowing size in input image	PSNR (dB)	MSE
Xiao et al. [7]	Median filter	3 × 3	30.69	0.9
		5 × 5	23.94	
		7 × 7	22.51	

Xiao et al. [7]	Mean filter	3 × 3	25.08	0.9
		5 × 5	21.68	
		7 × 7	20.16	

Xiao et al. [7]	Quantum inverse MFT filtering	3 × 3	35.69	1.4
		5 × 5	32.40	
		7 × 7	30.78	

Devakumari and Punithavathi [3]	Adaptive fuzzy median filter	3 × 3	33.60	1.3
		5 × 5	37.15	
		7 × 7	38.39	

Proposed method	QWTF	3 × 3	34.57	0.7
		5 × 5	38.41	
		7 × 7	43.50	

**Table 4:** Comparison between the proposed image segmentation method and other methods.

References	Accuracy (%)	Segmentation time (sec)
Abbass et al. [14]	92.78	10 to 60 sec for different images
Pereira et al. [15]	93.54	11.05
Moeskoops and Chen [20]	81	4
Cordeiro et al. [16]	92.50	2
El Adoui et al. [17]	98.50	4
Dalmıs et al. [19]	93.30	4
Milletari et al. [41]	82.39	4
Punitha et al. [23]	97.8	1.7
Mouelhi et al. [22]	98	2
Karabatak [27]	98.54	1
Rouhi et al. [24]	96.47	1.2
Proposed method	98.57	0.5

**Table 5:** The results of evaluation criteria for the proposed approach.

AUC	Sensitivity (%)	Feature rate (%)	Precision (%)	MSE	Dice similarity score (DSS) (%)
88.77	92.00	88.00	98.57	0.018	90.00

**Table 6:** The results of comparing the proposed approach with previous methods.

References	Precision (%)
Dehghan Khalilabad and Hassanpour [25]	95.45%
Kaymak et al., [26]	70.4%
Geweid and Abdallah [42]	85%
Karabatak [27]	98.54%
Wang et al. [28]	97.10
Rouhi et al. [24]	96.47%
Proposed method (Atrous pyramid CNN)	98.57%

## Data Availability

The mini-MIAS database of mammograms is available at https://peipa.essex.ac.uk/info/mias.html.
